# Modeling Various Survival Distributions using a Nonparametric Hypothesis Testing Based on Laplace Transform Approach with Some Real Applications

**DOI:** 10.1155/2022/5075716

**Published:** 2022-06-28

**Authors:** A. M. Gadallah, B. I. Mohammed, Abdulhakim A. Al-Babtain, Saima Khan Khosa, Mutua Kilai, M. Yusuf, M. E. Bakr

**Affiliations:** ^1^Department of Basic Sciences, Thebes Higher Institute for Engineering, Thebes Academy, Cairo, Egypt; ^2^Department of Mathematic. Faculty of Science, Al-Azhar University, First El Mokhaim El Madem St., Nasr City 11884, Cairo 11451, Egypt; ^3^Department of Statistics and Operation Research, College of Science, King Saud University, P.O. Box 2455, Riyadh 11451, Saudi Arabia; ^4^Department of Mathematics and Statistics University of Saskatchewan, Saskatoon, SK, Canada; ^5^Department of Mathematics, Pan African Insitute of Basic Science, Technology and Innovation, Nairobi, Kenya; ^6^Department of Mathematics, Helwan University, Cairo, Egypt; ^7^Department of Basic Sciences, Giza Higher Institute for Engineering and Technology, Cairo, Egypt

## Abstract

We hope to assess the different processing methodologies or the effectiveness of the devices or systems applied in this nonparametric statistical test by observing the failure behavior of the recorded survival data. The proposed second-order approach of new better than used (NBU 2) will be employed, which requires that the test data behaves either like NBU 2 property or exponentially. If the survival data is NBU 2, the proposed treatment method is likely to be beneficial. If the data are exponential, on the other hand, the recommended treatment method has no positive or negative influence on patients, as shown in the application section. To establish the validity of the test, we calculated the power of the proposed test and efficiency on both complete and censored data, compared the results to those of existing tests, and then applied the test to a range of real-world data.

## 1. Introduction

The estimation and testing of hypotheses were the two basic divisions of statistical inference. Generally, we have no idea what the true value of population parameters is. Thus, we have to estimate them. We do, however, have some theories concerning the true values of population parameters. The null hypothesis is frequently denoted by the sign H_0_, and the alternative hypothesis known as  H_1_. The null and alternative hypotheses must be defined prior to conducting any significant statistical test.

Various life distribution classes have been proposed during the last century to model various elements of aging. See, for example, the studies of Bakr et al. [1], Navarro and Pellerey [2], Bakr et al. [3], Navarro [4], Qureshi and Kumar [5], and Qureshi and Yusuf [6], for definitions and preservation of several classes of life distributions, such as IFR, NBU, UBA, UBAmgf, NBUE, and their duals.

The implications of the common classes, which include the majority of well-known classes such as IFR, NBU, NBUE, and HNBUE, are

(1) $$\begin{array}{c} \text{IFR}\Rightarrow \text{NBU}\Rightarrow \text{NBUE}\Rightarrow \text{HNBUE}. \end{array}$$

The survivor function is a base number that describes how long it takes for an event to occur.

The survivor function is defined as

(2) $$\begin{array}{c} {\bar{F}}_{t}\left(x\right)=\frac{\bar{F}\left(x+t\right)}{\bar{F}\left(t\right)},\;\bar{F}\left(t\right)>0. \end{array}$$

A fundamental property of surviving dissemination is the ability to age. The manuscript introduces a number of classes to categorize distributions.

The first aging is NBU. Here, *F*(*x*) has NBU property iff

(3) $$\begin{array}{c} \bar{F}\left(t\right)\;\bar{F}\left(x\right)\geq \bar{F}\left(t+x\right),\;\text{for all }t>0. \end{array}$$

The class NBUE distribution is the second aging class, and a life distribution has the NBUE property, represented by *X* ∈ NBUE iff

(4) $$\begin{array}{c} \int_{x}^{\infty }\bar{F}\left(u\right)du\leq \mu \;\bar{F}\left(x\right),\;\text{for all }x>0,\mu =E\left(X\right). \end{array}$$

**Definition 1 .**

A survival function $\bar{F}\left(x\right)$ considered NBU in the increasing concave order (*X* ∈ NBU(2)) iff

(5) $$\begin{array}{c} \int_{0}^{x}\bar{F}\left(u+t\right)du\leq \bar{F}\left(t\right)\int_{0}^{x}\bar{F}\left(u\right)du,\;\text{for all }x,t>0. \end{array}$$

The previous inequality has a physical meaning: in terms of rising concave ordering, the lifetime of a worn object with age *t* > 0 is stochastically shorter than that of a new one.

Barlow and Proschan [7], Abu-Youssef and Bakr [8], Abu-Youssef et al. [9], Franco et al. [10], Deshpande et al. [11], Hu and Xie [12], Qureshi and Yusuf [13], Hassan and Said [14], Sania Qureshi and Rashid Jan [15], Abu-Youssef et al. [16, 17], and Lia and Xie [18], and others proposed the probabilistic features of the aging distributions in the literature. The following are the relationships between the previous classes:

(6) $$\begin{array}{c} \text{NBUE}⊃\text{NBU }\left(2\right)⊃\text{NBU}. \end{array}$$

We have some genuine data in this research investigation, and we are trying to figure out whether H_0_: data is exponential or H_1_: data is NBU (2).

In this research study, we have got some real data, and we are trying to figure out whether H_0_: data is exponential or H_1_: data is NBU (2). To decide which H_0_ or H_1_ is true or to reach to a conclusion, we must first establish test statistics. The test statistic is a random variable that determines how closely a sample result matches one of these hypotheses under consideration.

Al-Gashgari et al. [19] and Gadallah [20] followed Atallah et al. [21] in developing a new approach of exponential testing that is more generic and flexible than goodness of fit.

This is how the research is structured: in Section 2, we produce a test statistic for the complete data using the Laplace transform approach. In Section 3, Monte Carlo null distribution critical points for data sets 5(5)100 are illustrated using Mathematica 8. For popular alternatives, Section 4 tabulates Pitman asymptotic efficiency, and Section 5 estimates the power of the test. In Section 6, a recommended test for appropriately filtered data is proposed. Finally, we discuss sets of medical real data in Section 7 to highlight the importance of our test.

## 2. Test Statistic for Complete Data

For *β*, *x* > 0, take *F*(*x*) = 1 − *e*^−*βx*^ , which is the exponential distribution class's distribution function *ξ*. Our formal objective is to compare *H*_0_ : *F* ∈ *ξ* and *H*_1_ : *F* ∈ NBU 2\*ξ*.

Lemma 2 provides a measure of deviation. As a result, it might be utilized to create a testing technique.

**Lemma 1 .**

If ∅(*s*) = *E*(*e*^−*sx*^), then

(7) $$\begin{array}{c} \delta =\frac{1}{s^{3}}\left[sE\left(x{\text{e}}^{-\text{sx}}\right)-\emptyset \left(s\right)\left(1-\emptyset \left(s\right)\right)\right]. \end{array}$$

**Proof**

Let us call the deviation from *H*_0_ the measure of departure as

(8) $$\begin{array}{c} \delta =\int_{0}^{\infty }\int_{0}^{\infty }\int_{0}^{x}\left[\bar{F}\left(t\right)\bar{F}\left(u\right)-\bar{F}\left(u+t\right)\right]e^{-s\left(x+t\right)}\;dudxdt=I-II, \end{array}$$

where

(9) $$\begin{array}{c} I=\int_{0}^{\infty }\int_{0}^{\infty }\int_{0}^{x}\bar{F}\left(t\right)\bar{F}\left(u\right)e^{-sx}e^{-st}\;dudxdt=\int_{0}^{\infty }\int_{x}^{\infty }e^{-su}\bar{F}\left(x\right)dudx\int_{0}^{\infty }E\left[I\left(X>t\right)\right]e^{-st}dt=\frac{1}{s^{3}}E^{2}\left[1-e^{-sx}\right]=\frac{1}{s^{3}}\left(1-2\emptyset \left(s\right)+\emptyset^{2}\left(s\right)\right),\\ II=\int_{0}^{\infty }\int_{0}^{\infty }\int_{0}^{x}\bar{F}\left(u+t\right)e^{-sx}e^{-st}\;dudxdt=\frac{1}{s^{3}}E\left[1-e^{-sx}-sxe^{-sx}\right]. \end{array}$$

Hence, the result follows.

We may derive the empirical estimator from (7) for *δ* as

(10) $$\begin{array}{c} {\hat{\delta }}_{n}=\frac{1}{s^{3}n\left(n-1\right)}\underset{i}{\sum }\underset{j}{\sum }\left\{sX_{i}e^{-{sX}_{i}}+e^{-{sX}_{i}}e^{-{sX}_{j}}-e^{-{sX}_{i}}\right\}. \end{array}$$

So, we can say that $\hat{\delta }$ is

(11) $$\begin{array}{c} {\hat{\delta }}_{n}=\frac{1}{s^{3}n\left(n-1\right)}\underset{i}{\sum }\underset{j}{\sum }\emptyset \left(X_{i},X_{j}\;\right), \end{array}$$

where

(12) $$\begin{array}{c} \emptyset \left(X_{i},X_{j}\;\right)=sX_{i}e^{-{sX}_{i}}+e^{-{sX}_{i}}e^{-{sX}_{j}}-e^{-{sX}_{i}}. \end{array}$$

The *U*-statistic theory can be used to obtain the limiting distribution of $\hat{\delta }\left(s\right)$.

Set

(13) $$\begin{array}{c} \emptyset \left(X_{1},X_{2}\right)=sX_{1}e^{-{sX}_{1}}+e^{-{sX}_{1}}e^{-{sX}_{2}}-e^{-{sX}_{1}}. \end{array}$$

Then,

(14) $$\begin{array}{c} E\left[\emptyset \left(X_{1},X_{2}\right)\left|X_{1}\right.\right]=sX_{1}e^{-{sX}_{1}}+\frac{1}{1+s}e^{-{sX}_{1}}-e^{-{sX}_{1}},\\ \text{E}\left[\emptyset \left(X_{1},X_{2}\right)\left|X_{2}\right.\right]=\frac{s}{1+s}+\frac{1}{1+s}e^{-{sX}_{2}}-\frac{1}{1+s}. \end{array}$$

Let

(15) $$\begin{array}{c} \xi \left(X\right)=E\left[\emptyset \left(X_{1},X_{2}\right)\left|X_{1}\right.\right]+E\left[\emptyset \left(X_{1},X_{2}\right)\left|X_{2}\right.\right]=sXe^{-sX}+\frac{1-s}{1+s}e^{-sX}-\frac{1}{{\left(1+s\right)}^{2}}. \end{array}$$

The asymptotic normality of the statistic (7) was demonstrated in Theorem 1.

**Theorem 1 .**

According to *U*-statistics theory, the statistic has the following characteristics:

(i) As *n*⟶∞, with mean of 0 and variance *σ*^2^, $\left({\hat{\delta }}_{n}-\delta \right)\;$ is asymptotically normal, such that
  (16) $$\begin{array}{c} \sigma^{2}=\text{Var}\left[\xi \left(X\right)\right]=E{\left(sXe^{-sX}+\frac{1-s}{1+s}e^{-sX}-\frac{1}{{\left(1+s\right)}^{2}}\right)}^{2} \end{array}$$
(ii) Under H_0_, the variance reduces to
  (17) $$\begin{array}{c} \sigma_{0}^{2}=\frac{s^{4}\left(1+2s\left(1+s\right)\right)}{{\left(1+s\right)}^{4}{\left(1+2s\right)}^{3}}. \end{array}$$

**Proof**

(i) We obtain the following results using U-statistic theory (Lee [22]):
  (18) $$\begin{array}{c} E\left[\xi \left(X\right)\right]=E\left(sXe^{-sX}+\frac{\left(1-s\right)}{\left(1+s\right)}e^{-sX}-\frac{1}{{\left(1+s\right)}^{2}}\right),\\ \sigma^{2}=\text{Var}\left[\xi \left(X\right)\right]=E{\left(sXe^{-sX}+\frac{\left(1-s\right)}{\left(1+s\right)}e^{-sX}-\frac{1}{{\left(1+s\right)}^{2}}\right)}^{2} \end{array}$$
(ii) In *H*_0_, it is obvious that *μ*_0_ = *E*[*ξ*(*X*)] = 0, and the variance is
  (19) $$\begin{array}{c} \sigma_{0}^{2}\left(s\right)=\frac{s^{4}\left(1+2s\left(1+s\right)\right)}{{\left(1+s\right)}^{4}{\left(1+2s\right)}^{3}}. \end{array}$$

## 3. Critical Points

Based on 10,000 simulated sample sizes *n* = 5 (5) 100 from the exponential distribution, we calculate the upper percentage points of the test statistic for our test in this section using Mathematica 8 Programming.

Table 1 shows a statistically significant percentile points at *s* = 0.4, 0.6.

Asymptotic normality improves, as the critical values decreases and their sample size increases, as in Table 1.

## 4. Pittman Efficiency

We can compare our test to the other courses to determine the quality of this procedure. Here, we choose the test *U*_*n*_ presented by Kayid et al. [23] and *δ*_*F*_*n*__^(2)^ presented by Mahmoud and Abdul Alim [24].

In this section, the PAE of our test is evaluated.

(20) $$\begin{array}{c} \text{PAE}\left(\delta \right)=\frac{{\left|\left(\partial /\partial \theta \right)\delta \right|}_{\theta ⟶\theta_{0}}}{\sigma_{0}}=\frac{1}{\sigma_{0}}\left|\frac{2}{s\left(s+1\right)}\int_{0}^{\infty }e^{-sx}\overset{¯}{F}\prime_{\theta_{0}}\left(x\right)dx-\frac{1}{s}\int_{0}^{\infty }xe^{-sx}\overset{¯}{F}\prime_{\theta_{0}}\left(x\right)dx\right|, \end{array}$$

where $\overset{¯}{F}\prime_{\theta_{0}}\left(x\right)={\left.\left(d/d\theta \right){\overset{¯}{F}}_{\theta }\left(u\right)\right|}_{\theta ⟶\theta_{0}}.$

Here, we use the following alternatives:

(i) Linear failure rate (LFR) family:
  (21) $$\begin{array}{c} {\bar{F}}_{1}\left(x\right)=e^{-x-\left(x^{2}/2\right)\theta },\;\theta ,x\geq 0. \end{array}$$
(ii) Weibull family:
  (22) $$\begin{array}{c} {\bar{F}}_{2}\left(x\right)=e^{-x^{\theta }},\;\theta \geq 1,x\geq 0. \end{array}$$
(iii) Makeham family:
  (23) $$\begin{array}{c} {\bar{F}}_{3}\left(x\right)=e^{-x-\theta \left(x+e^{-x}-1\right)},\;\theta ,x\geq 0. \end{array}$$

The null hypothesis H_0_ is attained at *θ* = 0 in (i) and (iii) and *θ* = 1 in (ii).

We investigate the PAE of our test *δ*, where

(24) $$\begin{array}{c} \text{PAE}\left(\delta ,\text{LFR}\right)=\frac{1}{\sigma_{0}\left(s\right)}\left|\frac{1}{s{\left(1+s\right)}^{4}}\right|,\\ \text{PAE}\left(\delta ,\text{Weibull}\right)=\frac{1}{\sigma_{0}\left(s\right)}\left|\frac{2}{s\left(1+s\right)}\int_{0}^{\infty }e^{-sx}\left(-xln\left(x\right)e^{-x}\right)dx-\frac{1}{s}\int_{0}^{\infty }e^{-sx}\left(-xln\left(x\right)e^{-x}\right)dx\right|,\\ \text{PAE}\left(\delta ,\text{Makeham}\right)=\frac{1}{\sigma_{0}\left(s\right)}\left|\frac{1}{s{\left(1+s\right)}^{2}{\left(2+s\right)}^{2}}\right|. \end{array}$$

Direct calculations of PAE of *U*_*n*_, *δ*_*F*_*n*__^(2)^, and *δ* at *s* = 0.4 and 0.6 are summarized in Table 2.

The PARE of *δ* with respect to *U*_*n*_ and *δ*_*F*_*n*__^(2)^ is shown in Table 3.

Tables 2 and 3 show the good performance of the selected families.

## 5. Estimates of Power

Table 4 illustrates the efficacy of the suggested test. For the LFR, Makeham, and Weibull distributions, these powers were estimated using 10,000 simulated samples with *n* = 10, 20, and 30 at a significance level of 0.05 (programming using Mathematica 8).

The suggested test has good validity for the Makeham and Weibull families and acceptable validity for the LFR family, as shown in Table 4.

## 6. Test Statistic for Censored Data

One of the most significant improvements in the life sciences has come from a property of survival data: if some of the participants did not observe the event of interest at the end of this research or at the time of analysis, the data is skewed. Some patients may still be alive or disease-free at the end of the experiment because the timing of survival or the end of disease is unknown. Individuals are referred to as censored observations or censored times when they cannot be followed up with after a research session.

In this section, a statistical test is developed to assess H_0_ and H_1_ with data that has been randomly right censored.

In the case of censored data, use Definition 1 and the Kaplan-Meier estimator; we can write the measure of departure as follows:

(25) $$\begin{array}{c} \delta_{c}=\frac{1}{s^{3}\left(n\right)\left(n-1\right)}\left[s\eta -\theta \left(1-\theta \right)\right], \end{array}$$

where

(26) $$\begin{array}{c} \theta =\int_{0}^{\infty }e^{-sx}dF\left(x\right),\\ \hat{\theta }=\overset{l}{\underset{m=1}{\sum }}e^{-sZ_{\left(m\right)}}\left(\overset{m-2}{\underset{p=1}{\prod }}C_{p}^{\delta_{p}}-\overset{m-1}{\underset{p=1}{\prod }}C_{p}^{\delta_{p}}\right),\\ \hat{\eta }=\overset{l}{\underset{j=1}{\sum }}\overset{j-1}{\underset{k=1}{\prod }}C_{m}^{\delta_{m}}\left(Z_{\left(j\right)}-Z_{\left(j-1\right)}\right). \end{array}$$

Table 5 shows a statistically significant percentile points of *δ*_*c*_ in (25), at *s* = 0.4, 0.6.

As shown in Table 5, the asymptotic normality improves, as the critical values decrease and their sample size increase.

## 7. Applications

We apply the conclusions in this work to certain real data sets to demonstrate their utility.

### 7.1. Application 1: A Case of Complete Data

**Example 1 .**

We apply the data presented in bakr et al. [1] (see Table 6), which represents the ages of the 40 patients with leukemia, taken in years.

In the two situations of $\hat{\delta }\left(0.4\right)$ and $\hat{\delta }\left(0.6\right)\;$ as *n* = 40, we calculate the statistics in (7): $\hat{\delta }\left(0.4\right)=1.5$ and $\hat{\delta }\left(0.6\right)=0.43$, both of which are above the critical value of Table 1. Consequently, the data set has the property of NBU (2).

**Example 2 .**

Consider the data in Bakr et al. [3] (see Table 7), which represent 39 liver cancer patients taken from El-Minia Cancer Center, Ministry of Health, Egypt, which entered in 1999.

In the two situations of $\hat{\delta }\left(0.4\right)$ and $\hat{\delta }\left(0.6\right)\;$ as *n* = 39, we calculate the statistics in (7): $\hat{\delta }\left(0.4\right)=0.07$ and $\hat{\delta }\left(0.6\right)=0.003$, both of which are under the critical value of Table 1. Consequently, the data set has no property of NBU (2).

### 7.2. Application 2: A Case of Censored Data

**Example 3 .**

We use data from Mahmoud et al. [25] (see Tables 8 and 9) to represent the age (in days) of 51 liver cancer patients from the Egyptian Ministry of Health's Elminia Cancer Center who began medical examinations in 2000. (1999). Only 39 patients are included in the study (right-censored), while the other 12 are excluded (missing from the study). Tables 8 and9show the list of ordering information.

In the two situations of$\;{\hat{\delta }}_{c}\left(0.4\right)$ and $\;{\hat{\delta }}_{c}\left(0.6\right)$ as *n* = 51, we calculate the statistics in (25): $\;{\hat{\delta }}_{c}\left(0.4\right)=1.6\times 10^{70}$ and $\;{\hat{\delta }}_{c}\left(0.6\right)=3.88\times 10^{68}$, both of which are above the critical value of Table 5. Consequently, the data set has the property of NBU (2).

**Example 4 .**

Consider the survival intervals in weeks reported by Lee and Wolfe [26] (see Tables 10 and 11) for 61 patients with unresectable lung cancer who were treated with cyclophosphamide. There are 33 uncensored observations and 28 censored observations for patients whose therapy was terminated owing to an evolving condition.

In the two situations of $\;{\hat{\delta }}_{c}\left(0.4\right)$ and $\;{\hat{\delta }}_{c}\left(0.6\right)$ as *n* = 61, we calculate the statistics in (25): $\;{\hat{\delta }}_{c}\left(0.4\right)=5.07\times 10^{14}$ and $\;{\hat{\delta }}_{c}\left(0.6\right)=1.31\times 10^{14}$, both of which are above the critical value of Table 5. Consequently, the data set has the property of NBU (2) Table 12 show the notations and abbreviations.

## 8. Conclusion

We devised a statistical testing approach (Laplace transform technique) for the largest class of life distribution NBU (2) in both complete and censored data to aid in the quality assessment of prospective cancer therapies. Our testing revealed whether the suggested therapies had a good or negative influence on patient survival as shown in the four discussed examples. The effectiveness of the suggested statistical test was computed and compared to existing tests to confirm that it produced good findings. Regardless of the kind of treatment technique, the suggested test can be used to evaluate the efficacy of any treatment strategy in any field of medical study. This test, however, should not be used to compare two distinct treatment options.

On the other hand, the efficiency of our proposed tests is compared to the tests of Kayid et al. [14] and *δ*_*F*_*n*__^(2)^ presented by Qureshi and Jan [15], which are based on Pitman's asymptotic relative efficiency and employ several well-known life distributions, namely, the LFR and the Weibull family. Finally, the paper's findings are tested using actual real-world data.

## Figures and Tables

**Table 1:** The percentile points of ${\hat{\delta }}_{n.}$

${\hat{\delta }}_{n};s=0.4$				${\hat{\delta }}_{n};s=0.6$		
*n*	95%	98%	99%	95%	98%	99%
5	0.882897	1.17189	1.38849	0.396275	0.502898	0.562419
10	0.525925	0.667885	0.752876	0.221699	0.274836	0.299154
15	0.388132	0.486231	0.556578	0.166089	0.206706	0.234874
20	0.323144	0.413406	0.467084	0.145573	0.178422	0.196138
25	0.28863	0.350084	0.39139	0.122991	0.150936	0.169784
30	0.258019	0.320188	0.365255	0.10865	0.138144	0.166397
35	0.235234	0.293309	0.331031	0.105987	0.127848	0.14191
40	0.215066	0.265283	0.295422	0.0950951	0.129734	0.141408
45	0.206855	0.25257	0.284129	0.0873638	0.115054	0.125216
50	0.191667	0.235837	0.270402	0.0871117	0.108423	0.121646
55	0.18134	0.226473	0.256603	0.0790283	0.10263	0.118798
60	0.172598	0.213932	0.244309	0.073819	0.093089	0.0996918
65	0.165691	0.204694	0.235163	0.0700623	0.082458	0.101185
70	0.158049	0.195075	0.213855	0.0725355	0.0930558	0.100772
75	0.154806	0.188446	0.212941	0.0691197	0.083419	0.0928818
80	0.151963	0.185998	0.212013	0.065666	0.0828855	0.0962278
85	0.143606	0.178592	0.201549	0.0645971	0.075949	0.0900691
90	0.137717	0.173923	0.199664	0.0645374	0.076169	0.0858537
95	0.137395	0.169832	0.194102	0.0621102	0.077558	0.0897414
100	0.134282	0.162602	0.184573	0.0613547	0.0794837	0.0925321

**Table 2:** PAE of *U*_*n*_, *δ*_*F*_*n*__^(2)^, and *δ*.

Distribution	*U*_*n*_	*δ*_*F*_*n*__^(2)^	*δ*(0.4)	*δ*(0.6)
LFR	0.5809	0.217	3.35	3.40
Weibull	2.3238	0.050	2.16	2.28
Makeham	0.2585	0.144	1.47	1.50

**Table 3:** Relative efficiency of *δ* with respect to *U*_*n*_ and *δ*_*F*_*n*__^(2)^.

Distribution	*e*(*δ*(0.4), *U*_*n*_)	*e*(*δ*(0.6), *U*_*n*_)	*e*(*δ*(0.4), *δ*_*F*_*n*__^(2)^)	*e*(*δ*(0.6), *δ*_*F*_*n*__^(2)^)
LFR	5.76	5.85	15.2	15.67
Weibull	0.93	0.98	43.20	45.6
Makeham	5.69	5.80	10.2	10.41

**Table 4:** The powers at *α* = 0.05.

Distribution	*n*	*θ* = 2	*θ* = 3	*θ* = 4
LFR	10	0.504	0.573	0.663
	20	0.519	0.613	0.717
	30	0.520	0.643	0.744
Makeham	10	0.832	0.900	0.925
	20	0.956	0.999	1
	30	1	1	1
Weibull	10	0.753	0.821	0.915
	20	0.838	0.995	1
	30	0.999	1	1

**Table 5:** The upper percentile points of ${\hat{\delta }}_{\text{c}}$.

${\hat{\delta }}_{c}\left(0.4\right)$				${\hat{\delta }}_{c}\left(0.6\right)$		
*n*	95%	98%	99%	95%	98%	99%
2	0.535606	0.583176	0.61155	0.007199	0.0296232	0.0501468
4	0.0985967	0.106324	0.109739	0.00717465	0.00973058	0.0118462
6	0.0382919	0.0418751	0.0429949	0.00292626	0.00471896	0.00502581
8	0.0220675	0.0235447	0.0241831	0.00186656	0.0023683	0.00269643
10	0.0138634	0.0147497	0.0150687	0.0012502	0.00168057	0.00182981
12	0.00944369	0.00992625	0.010188	0.00073221	0.00102515	0.00114684
14	0.00667813	0.0071701	0.00738161	0.00035340	0.00072136	0.00083496
16	0.00489464	0.00550842	0.00565949	0.00018206	0.00041354	0.00061089
18	0.00372462	0.00419779	0.00434607	0.00003021	0.00026197	0.00041052
20	0.00266338	0.00307783	0.00332981	0.0000427	0.00015384	0.00029494

**Table 6:** 

0.315	0.496	0.616	1.145	1.208	1.263	1.414	2.025	2.036	2.162
2.211	2.370	2.532	2.693	2.805	2.910	2.912	3.192	3.263	3.348
3.348	3.427	3.499	3.534	3.767	3.751	3.858	3.986	4.049	4.244
4.323	4.381	4.392	4.397	4.647	4.753	4.929	4.973	5.074	4.381

**Table 7:** The periods of orderly life (in days).

10	14	14	14	14	14	15	17	18	20
20	20	20	20	23	23	24	26	30	30
31	40	49	51	52	60	61	67	71	74
75	87	96	105	107	107	107	116	150	

**Table 8:** Noncensored data.

10	14	14	14	14	14	15	17	18	20
20	20	20	20	23	23	24	26	30	30
31	40	49	51	52	60	61	67	71	74
75	87	96	105	107	107	107	116	150	

**Table 9:** Censored data.

30	30	30	30	30	60	150	150	150	150
150	185								

**Table 10:** Noncensored data.

0.43	2.86	3.14	3.14	3.43	3.43	3.71	3.86	6.14	6.86	9.00
9.43	10.71	10.86	11.14	13.00	14.43	15.71	18.43	18.57	20.71	29.14
29.71	40.57	48.57	49.43	53.86	61.86	66.57	68.71	68.96	72.86	72.86

**Table 11:** Censored data.

0.14	0.14	0.29	0.43	0.57	0.57	1.86	3.00	3.00	3.29	3.29
6.00	6.00	6.14	8.71	10.57	11.86	15.57	16.57	17.29	18.71	21.29
23.86	26.00	27.57	32.14	33.14	47.29					

**Table 12:** Notations and abbreviations.

IFR	Increasing failure rate
NBU	New better than used
NBU 2	New better than used in the second order
NBUE	New better than used in expectation
HNBUE	Harmonic new better than used in expectation
NBUCL	New better (worse) than used in a convex Laplace ordering
UBAL	Used better than age in Laplace transform
UBA_mgf_	Used better than age in moment generating function

## Data Availability

The data are mentioned along the paper.
